This article has been retracted.

# Correlation of Serum Chemokine (C-C Motif) Ligand 21 and Heat Shock Protein 90 with Preeclampsia

**DOI:** 10.1155/2022/2156424

**Published:** 2022-08-03

**Authors:** Weina Yang, Xuemei Yang, Su'e Zhang, Limei Zhang, Wenze Wang, Li Wang

**Affiliations:** Obstetrics Department, Shijiazhuang Obstetrics and Gynecology Hospital, Key Laboratory of Maternal and Fetal Medicine of Hebei Province, Shijiazhuang, Hebei, China

## Abstract

**Objective:**

The study aimed to explore the correlation of serum chemokine (C-C motif) ligand 21 (CCL21) and heat shock protein 90 (Hsp90) with preeclampsia (PE).

**Methods:**

Between June 2021 and June 2022, 50 pregnant women with PE were included in the PE group, and 50 healthy pregnant women were included in the control group. The serum levels of CCL21 and Hsp90 were compared between the two groups.

**Results:**

PE patients showed significantly higher levels of CCL21 and Hsp90 than healthy pregnant women (*P* < 0.05). Correlation analysis showed a positive correlation between CCL21 and Hsp90 levels (*r* > 0, (*P* < 0.05)). Binary logistic regression analysis suggested that high expression of CCL21 and Hsp90 were influencing factors for PE (OR >1, (*P* < 0.05)). The area under the receiver operating characteristic (AUC) curves of Hsp90 and CCL21 levels for predicting PE were 0.895 and 0.864, respectively, suggesting a good predictive value.

**Conclusion:**

Serum CCL21 and Hsp90 show great potential as disease markers for PE prediction. Further trials are, however, required prior to clinical promotion.

## 1. Introduction

Preeclampsia (PE) is a severe hypertensive disorder of pregnancy, which is manifested by hypertension, edema, proteinuria, and dysfunction of the heart and other organs, and is a major cause of maternal mortality [1]. The pathogenesis of PE is closely associated with placental ischemia and vascular endothelial damage. PE develops with abnormal trophoblast function in the mother, impaired physiological processes in the intrauterine spiral arteries, and damaged vascular endothelial cells [2]. In recent years, the prevalence of adverse pregnancies has been increasing, with hypertension, obesity, and higher age as potential influencing factors for adverse pregnancies [3]. The treatment of PE mainly focuses on the regulation of maternal blood pressure, blood circulation improvement, and complication prevention, and commonly used drugs include magnesium sulfate and nifedipine [4]. PE belongs to the category of “epilepsy” in traditional Chinese medicine (TCM) and is caused by spleen deficiency, kidney yang deficiency, essence and blood deficiency, and liver yang hyperactivity. In TCM, PE is mostly treated by “tonic for deficiencies and elimination for excesses” to manage disease development and improve patient prognosis [5, 6].

Heat shock proteins (Hsps) are a class of cellular chaperone proteins that are produced by biological cells following stressor stimulation [7]. Clinical research has found that the level of heat shock proteins in the body of patients with cardiovascular disease is closely related to the severity of the disease [8]. Hsp90 plays an important role in cell growth and development, differentiation, and protection of cells under stressful conditions [9]. As small molecules secreted proteins, chemokines enable cells to undergo chemotactic movements to participate in inflammatory and immune responses [10]. Chemokine (C-C motif) ligand 21 (CCL21) is secreted by activated T-lymphocytes and endothelial cells and is involved in humoral immunity to promote inflammatory responses [11].

Currently, PE management emphasizes early diagnosis and symptomatic treatment, and screening for high-risk factors and establishing accurate prediction methods contribute positively to the prognosis of PE [12, 13]. Thus, the present study was undertaken to explore the correlation of serum CCL21 and Hsp90 with PE.

## 2. Materials and Methods

### 2.1. Patient Characteristics

Between June 2021 and June 2022, 50 pregnant women with PE were included in the PE group, and 50 healthy pregnant women were included in the control group. All patients provided written informed consent, and the experiment was undertaken as per the Declaration of Helsinki ethical guidelines for clinical research (ethical approval number: XD-GXQ20200703). The patient characteristics of the two groups were comparable (*P* > 0.05) (Table 1).

### 2.2. Inclusion and Exclusion Criteria

#### 2.2.1. Inclusion Criteria

Patients with a singleton pregnancy, without a history of chronic medical conditions, with confirmed PE as per the American College of Obstetricians and Gynecologists (ACOG) guidelines [10], with normal prepregnancy blood pressure, 24 h proteinuria ≥300 mg, protein/creatinine ≥0.3 mg/dL, urinary protein ≥++, and proteinuria (−), and with thrombocytopenia, renal insufficiency, impaired liver function, pulmonary edema, and new onset headache were included.

#### 2.2.2. Exclusion Criteria

Patients with medical or surgical diseases, with multiple pregnancies or fetal developmental malformations, who underwent artificial insemination or in vitro fertilization, without blood sample cryopreservation in early pregnancy, or who were lost during maternity examination were excluded.

### 2.3. Determination of CCL21 and Hsp90 Levels

3–5 mL of maternal peripheral blood was collected at 11–13 weeks of gestation and stored in a −80°C refrigerator for the following assays. The expression levels of CCL21 and Hsp90 in peripheral blood of pregnant women in early pregnancy were determined by quantitative real-time fluorescence PCR (qRT-PCR). The assay instrument is the American Bio-tech automatic enzyme standard instrument with a detection wavelength of 450 nm, and the kit is produced by Shanghai Enzyme Link Biological Co. Ltd.

### 2.4. Statistical Analysis

SPSS 23.0 software was used for data analyses. Count data were expressed as *n* (%) and analyzed using the chi-square test. The correlation of serum CCL21 and Hsp90 was analyzed by bivariate Pearson linear correlation analysis. The analysis of the effect of CCL21 and Hsp90 on PE was performed by the logistic regression analysis test and the receiver operating curve (ROC) was plotted to test the value of CCL21 and Hsp90 for predicting PE. *P* < 0.05 was used as a cutoff value for statistical significance.

## 3. Results

### 3.1. Serum Levels of CCL21 and Hsp90

PE patients showed significantly higher serum levels of CCL21 and Hsp90 than healthy pregnant women (*P* < 0.05) (Table 2).

### 3.2. Correlation between CCL21 and Hsp90

Bivariate Pearson linear correlation analysis demonstrated a positive correlation between serum CCL21 and Hsp90 levels in PE patients (*r* = 0.510, *P* < 0.001). (Figure 1).

### 3.3. Effect of Serum CCL21 and Hsp90 on PE

The baseline data and serum CCL21 and Hsp90 were used as covariates, PE was the dependent variable (1 = combined, 0 = uncombined), and a multiple regression model was established after binary logistic regression analysis. After preliminary binary regression analysis and calibration for mutual effects between individual data, serum CCL21 and Hsp90 overexpression were indicated as influential factors for PE (OR > 1, *P* < 0.05). (Table 3).

### 3.4. Predictive Value of Serum CCL21 and Hsp90 for PE

CCL21 and Hsp90 levels were used as test variables for all participants and whether PE was combined or not was used as a status variable (1 = combined, 0 = not combined). The ROC curve (Figure 2) analysis showed that the AUCs of serum CCL21 and Hsp90 levels for predicting PE risk were 0.895 and 0.864, respectively. The corresponding optimal threshold, specificity, sensitivity, and Jorden index for each index are shown in Table 4.

## 4. Discussion

Without proper treatment, PE may lead to maternal hypertension, proteinuria, hepatic, and renal insufficiency that eventually cause intrauterine hypoxia and growth restriction in the fetus and increase the risk of cardiovascular disease [14]. The complex etiology of PE involves immune system dysfunction, inflammatory cytokines, and hormonal abnormalities, in which the activation of significant numbers of inflammatory cells in vivo damages the vascular endothelium, leading to abnormal vascular remodeling and the development of PE [15]. The current treatment for PE focuses on regulating blood pressure, improving blood circulation, and preventing complications. Nifedipine extended-release tablets dilate systemic blood vessels and relax smooth muscle by inhibiting calcium ion inward flow and also prevent preterm abortion [16]. Magnesium sulfate prevents preterm labor by antagonizing calcium ions to inhibit uterine contractions, and magnesium ions act directly on vascular smooth muscle to normalize the blood pressure [17].

In TCM, the etiology of PE is attributed to internal movement of liver wind, phlegm, and fire, deficiency of kidney essence, loss of nourishment of the heart and liver, hyperactivity of liver yang into the fire, internal heat from yin deficiency, scorching of fluid into phlegm, mutual knotting of phlegm and heat, deficiency of the spleen and dampness, and heat from depression. Qiju Dihuang decoction is commonly used clinically to treat PE by nourishing yin, calming the wind, pacifying the liver, and subduing yang [18, 19]. Because the inflammatory response in the early stages of PE elicits alterations in the levels of numerous serum markers before the emergence of clinical symptoms, the screening for early predictors of PE development and early intervention in the treatment of PE is of great importance [20].

The results of the present study showed that PE patients had significantly higher serum levels of CCL21 and Hsp90, suggesting the association of the abnormal expression of CCL21 and Hsp90 with PE development. CCL21 is mainly distributed in the peripheral immune organs and tissues and chemotaxis of various immune cells. Numerous related reports have shown that CCL21 contributes to the production of a large number of inflammatory cells such as a tumor necrosis factor and interleukin-8, thereby triggering inflammatory responses and aggravating the disease [21]. Hsp90, a marker of PE, is usually considered an intracellular protein with molecular chaperone and cytoprotective functions that protects cells from apoptosis, and elevation in its level indicates a risk of the nonphysiological state that triggers an immune response [22]. Studies have confirmed that Hsp90 functions as a proangiogenic agent, especially during embryogenesis, and binds to VEGFR-1 and displaces VEGF, prompting VEGFR-2 activation and intermolecular transphosphorylation and causing endothelial dysfunction after amplified angiogenesis, which is a common manifestation of PE [23]. In addition, clinical studies have revealed that Hsp family analogs exert a variety of biological functions such as molecular chaperones, antioxidant, antiapoptotic, proliferation-promoting, and stress-tolerant cells by binding to substrate proteins [24]. All these results are similar to the results of the present study and reinforce the credibility of our conclusions.

Logistic regression analysis showed that high expressions of serum CCL21 and Hsp90 were influencing factors of PE, and the ROC curve found that the AUCs of CCL21 and Hsp90 for predicting PE were 0.897 and 0.862, respectively, suggesting a favorable predictive value. This result also supported our hypothesis. Thus, CCL21 and Hsp90 may be involved in the development of PE and show good potential to assess the disease conditions of PE. In addition, correlation analysis revealed a positive correlation between CCL21 and Hsp90 levels, suggesting that serum CCL21 and Hsp90 in PE patients interact with each other and participate in the pathogenesis of PE.

Immunologically, the embryo must rely on the immune tolerance balance between the mother and the fetus to attach to the uterus and survive until delivery, and disruption of this balance results in pathological pregnancy [25]. A large body of evidence suggests an association between the development of PE and an imbalance of maternal immune tolerance. Hsp plays a key role in the regulation of tumor cell differentiation and apoptosis [26]. Hsp90 is one of the most active molecular chaperone proteins in cells and is involved in responses in multiple signaling pathways that affect cell growth and development, differentiation, and protein synthesis [27, 28]. The limitations of the present study lie in the small sample size and the absence of long-term follow-up. Future multicenter studies with a larger sample size will be conducted to provide more reliable clinical data.

## 5. Conclusion

Serum CCL21 and Hsp90 show great potential as disease markers for PE prediction. Further trials are, however, required prior to clinical promotion.

## Figures and Tables

**Figure 1:** Correlation between CCL21 and Hsp90.

**Figure 2:** ROC curves of serum CCL21 and Hsp90 for predicting PE.

**Table 1:** Patient characteristics.

	PE	Control	*t*/*Z*	*P* value
*n*	50	50		
Age (years)	30.24 ± 4.17	29.68 ± 3.41	1.452	0.2122
BMI (kg/m^2^)	21.66 ± 3.11	21.22 ± 2.67	0.947	0.4523
Gestational week (weeks)	38.68 (37.74∼39.41)	39.43 (38.86∼40.05)	3.327	<0.001
Proteinuria (*g*/24 h)	0.42 ± 0.34	0.00	5.328	<0.001
Systolic blood pressure (mmHg)	141.5 (131.32∼143.82)	127.00 (112.00∼124.00)	6.424	<0.001
Diastolic blood pressure (mmHg)	95.52 (91.35∼104.45)	78.00 (73.00∼83.00)	6.657	<0.001

**Table 2:** Serum levels of CCL21 and Hsp90 ($\bar{x}$ ± *s*).

Group	*n*	Hsp90	CCL21
PE	50	94.56 ± 29.30	289.15 ± 54.32
Control	50	24.65 ± 15.11	168.45 ± 31.23
*χ * ^2^/*t*		9.8762	18.820
*P* value		<0.001	<0.001

**Table 3:** Effect of serum CCL21 and Hsp90 on PE.

Variables	B	S.E	Wals	*P*	OR value
Constants	8.237	1.536	56.324	<0.001	0.000
Age	0.378	0.584	0.713	0.654	1.433
CCL21	1.146	0.016	60.423	<0.001	1.212
Hsp90	3.023	0.687	53.412	<0.001	1.847

**Table 4:** Predictive value of serum CCL21 and Hsp90 for PE.

Indices	CCL21	Hsp90
AUC	0.864	0.895
95%CI	0.808∼0.918	0.843∼0.942
Standard error	0.031	0.027
*P* value	<0.001	<0.001
Optimal threshold	301.203 pg/mL	137.256 ng/mL
Specificity	0.958	0.976
Sensitivity	0.892	0.873
Jorden index	0.845	0.844

## Data Availability

No data were used to support this study.
